RETRACTED

# Formation of Proto-Kranz in C3 Rice Induced by Spike-Stalk Injection Method

**DOI:** 10.3390/ijms22094305

**Published:** 2021-04-21

**Authors:** Dexing Jiang, Feng Wang, Haizi Zhang, Wenwen Gao, Xi Tong, Chuangen Lv, Guoxiang Chen

**Affiliations:** 1 Jiangsu Key Laboratory of Biodiversity and Biotechnology, College of Life Sciences, Nanjing Normal University, Nanjing 210023, China; dxjiang0525@163.com (D.J.); 17805003839@163.com (F.W.); zhanghaizi@163.com (H.Z.); 15735642030@163.com (W.G.); 15651765792@189.com (X.T.); 2 Sino-Canada International School, Suzhou 215200, China; 3 Institute of Food Crops, Jiangsu Academy of Agricultural Sciences, Nanjing 210014, China

**Keywords:** C4 rice, proto-Kranz, photosynthetic efficiency, crop improvement, spike-stalk injection

## Abstract

Introduction of C4 photosynthetic traits into C3 crops is an important strategy for improving photosynthetic capacity and productivity. Here, we report the research results of a variant line of sorghum–rice (SR) plant with big panicle and high spikelet density by introducing sorghum genome DNA into rice by spike-stalk injection. The whole-genome resequencing showed that a few sorghum genes could be integrated into the rice genome. Gene expression was confirmed for two C4 photosynthetic enzymes containing pyruvate, orthophosphate dikinase and phosphoenolpyruvate carboxykinase. Exogenous sorghum DNA integration induced a series of key traits associated with the C4 pathway called “proto-Kranz” anatomy, including leaf thickness, bundle sheath number and size, and chloroplast size in bundle sheath cells. Significantly, transgenic plants exhibited enhanced photosynthetic capacity resulting from both photosynthetic CO_2_-concentrating effect and improved energy balance, which led to an increase in carbohydrate levels and productivity. Furthermore, such rice plant exhibited delayed leaf senescence. In summary, this study provides a proof for the feasibility of inducing the transition from C3 leaf anatomy to proto-Kranz by spike-stalk injection to achieve efficient photosynthesis and increase productivity.

## 1. Introduction

C4 photosynthesis evolved from the original C3 pathway during a global decline in atmospheric CO_2_ levels [1]. Despite its biochemical and anatomical complexity, C4 photosynthesis at least 66 times emerged independently in different plant families in approximately 18 lineages. C3 plants, which fix atmospheric CO_2_ to the 3-phosphoglycerate (3-PGA) compound for carbon fixation through Calvin cycle by Rubisco, are the most abundant crops and provide the most dietary calories to human diets [2]. In comparison with the ancestral C3 pathway, C4 plants form a special carbon shuttle system called C4 pathway, in which carbon is first fixed by incorporating CO_2_ into a four-carbon compound oxaloacetate (OAA) and then converted to the transport metabolites malate or aspartate [3]. This special carbon shuttle largely lowers rates of photorespiration and increases the efficiency of photosynthesis by facilitating a high CO_2_/O_2_ ratio at the site of Ribulose-bis-phosphate carboxylase/oxygenase (Rubisco) [4]. C4 photosynthesis confers improved radiation, nitrogen, and water-use efficiencies relative to C3 plants while reducing photorespiration to a minimum in severe environments, such as hot, arid, and saline areas [5]. With the prominent changes of global climate and the rapid increase of the world’s population, it has been proposed to improve photosynthetic efficiency by changing the types of photosynthetic pathway that is utilized or by optimizing the components of an existing pathway as a feasible way to enhance the yield potential of major crops [5,6,7].

RETRACTED

Many attempts have been made to integrate traits of C4 photosynthesis into C3 crops, which has the potential to greatly increase the yields of C3 crops [8]. One of the major challenges in this research field is to introduce Kranz anatomy into C3 plant leaves. In both monocots [9] and eudicots [10,11,12], proto-Kranz anatomy is characterized by increased organelle volume in the vascular sheath cells around the leaf vasculature, with chloroplasts accumulating the photosynthetic enzyme Rubisco and mitochondria accumulating the photorespiratory enzyme glycine decarboxylase. In the grasses, most of the C4 origins are grouped into the “PACMAD” clade [13]. Rice belongs to the BEP clade, which is not featured in any C4 taxa. Rice leaf possesses multiple anatomical features that are intermediate to C4 grasses, such as an analogous mesophyll thickness [14], an intermediate ratio of mesophyll to bundle sheath cells [15], the concentric arrangement of disklike-shaped mesophyll cells around a vascular bundle sheath [16], and a modest number of well-developed chloroplasts in the bundle sheath cells [14,15]. Therefore, a rational first step to engineering C4 rice is to induce proto-Kranz by activating organelle biogenesis in bundle sheath cells.

A new method of gene transformation is first reported for transforming exogenous DNA into cereal plants by Pena et al. [17]. On the basis of Pena’s method, Zhao et al. [18] further modified this technique called spike-stalk injection, in which the exogenous DNA was injected into the uppermost internode of a rice stem when the recipient rice had undergone meiosis. Hu et al. [19] recently reported that the spike-stalk injection method could cause extensive phenotypic and genotypic variations for rice by genomewide comparison, and preliminary results confirmed that some special DNA fragments from *Oryza eichingeri* were integrated in the rice RH78 genome. Spike-stalk injection can overcome the interspecific crossing barriers between different species during chromosome pairing. In the current study, such a variant rice line, so-called sorghum–rice (SR) with big panicle and high spikelet density, was obtained through the introduction of the sorghum genome DNA into rice by spike-stalk injection. Therefore, the objective of this study was to explore whether the treatment of spike-stalk injection can integrate some photosynthetic traits of sorghum (C4 plant) into rice (C3 plant).

RETRACTED

## 2. Results

### 2.1. Genome Resequencing of Rice SR

Whole-genome resequencing of transgenic rice SR yielded 25.78 Gb of raw sequencing data, and 25.38 Gb clean data were retained for downstream analysis after a series of corrections and filters (Table S1). The clean data were then aligned to the high-quality *indica* rice R498 genome and sorghum BTx623 genome using the Burrows–Wheeler Aligner (BWA). In total, 158,047,250 and 174,529 high-quality reads were generated from the *indica* rice R498 genome and sorghum BTx623 genome, respectively, among which 149,439,894 (94.55%) and 124,282 (71.21%) reads were uniquely and confidently mapped to the reference genome, indicating that a small number of sorghum genes can be integrated into the rice genome by spike-stalk injection (Table S1, Figure 1A). Since sorghum belongs to a typical C4 plant, we hypothesized that the introduction of exogenous sorghum DNA may induce the expression of C4 photosynthetic enzymes in rice SR. To verify this hypothesis, we detected the mRNA levels encoding sorghum C4 photosynthetic enzymes (PEPC, PEPCK, PPDK, and NADP-ME). However, only the expression of *SbPEPCK* and *SbPPDK* was detected in SR (Figure 1B).

### 2.2. Increased Vegetative Biomass in Rice SR

Significant differences between wild type (WT) and SR plants were observed in plant development or phenotype under normal conditions (Figure 2 and Figure S1). SR exhibited a more developed root system and larger stem diameter. The plant height was increased significantly in SR compared with WT (Figure 2C), whereas tiller number was decreased (Figure 2E). The flag leaf length (Figure 2F), width (Figure 2G), and area (Figure 2H) of SR were also significantly greater than those of WT (Figure 2B). In addition, relative to WT, SR had delayed leaf yellowing after flowering, which may lead to an increase in several agronomic traits. Collectively, these differences translated into a significant increase in total dry weight for SR (Figure 2D).

RETRACTED

### 2.3. Proto-Kranz Anatomy and Delayed Leaf Senescence in Rice SR

To determine whether the proto-Kranz anatomy is induced by the introduction of exogenous sorghum DNA in rice, we measured the changes of transgenic rice leaf structures (Figure 3). The number of rice SR bundle sheaths (BSs) including large bundle sheaths (LBSs) and small bundle sheaths (SBSs) was significantly increased relative to wild type, but the interbundle sheath distance was also increased (Figure 3A−E). By observing the cross sections of the central parts of flag leaves, it was found that SR increased leaf thickness at both large bundle sheaths (LBSs) and small bundle sheaths (SBSs), and increased bundle sheath (BS) size, and retained more Chl content (Figure 3F). Transmission electron microscopy (TEM) analysis was conducted to reveal the changes in the chloroplast morphology and structure in bundle sheath cells (BSCs) and mesophyll cells (MCs) of WT and SR (Figure 3G,H). Compared with that in WT, the size of chloroplast was dramatically increased in BSCs of SR (Figure 3G). In addition, at 14 DAF, the chloroplasts of SR were intact with highly stacked grana thylakoids, and the grana structure remained intact, whereas WT showed a severe dismantling of grana thylakoids, less starch grain, and a large number of osmiophilic plastoglobules (Figure 3G,H). Collectively, these results indicate that the introduction of exogenous sorghum DNA into rice can induce the formation of proto-Kranz anatomy, recapitulating one of the earliest steps in C4 evolution.

### 2.4. Increased Photosynthetic Capacity in Rice SR

Photosynthesis is an important factor in determining crop yield. To evaluate whether photosynthetic capacity was enhanced in the transgenic rice SR, the flag leaf photosynthesis of SR in response to different light levels was compared with WT with the same set of plants at 7 DAF growth stage. As shown in Figure 4A, only small differences in photosynthetic rate were observed between WT and SR when photon flux density (PFD) was less than 200 μmol m^−2^ s^−1^, whereas the differences were much more pronounced at saturated PFDs. Furthermore, light-saturated photosynthetic rate (A_max_) and apparent quantum yield (AQY) values were significantly increased by 26.2% and 29.9% (Figure 4B,C), respectively. During the postflowering stage, the flag leaves of SR retained much higher chlorophyll (Chl) levels, while the WT leaves showed a significant decrease in Chl levels (Figure 4D). As a result, the Chl content of SR was 76.9% higher than that of WT at 28 DAF (Figure 4D). To further examine the photosynthetic performance of SR during natural senescence, we measured the photosynthetic rate, F_v_/F_m_ ratio (maximum quantum efficiency of photosystem II), and total performance index (PI_total_). The results demonstrated that all these parameters in the WT and SR flag leaves became progressively lower, with that in WT decreasing even more rapidly (Figure 4E−G). Notably, the photosynthetic rate and PI_total_ of SR were consistently higher than those of WT after flowering (Figure 4E,G). Together these results demonstrate that the introduction of exogenous sorghum DNA enhances the photosynthetic capacity in rice.

RETRACTED

### 2.5. Reduced ROS Accumulation and Oxidative Damage in the Leaves of Rice SR during Natural Senescence

As it is well known, the generation of reactive oxygen species (ROS) is one of the earliest responses of plant leaf senescence, which prompted us to investigate the accumulation of ROS in SR during natural senescence. At 7 DAF, the O_2_^–^ and H_2_O_2_ levels in the WT leaves were slightly higher than those in SR. However, both O_2_^–^ and H_2_O_2_ were significantly reduced in the SR leaves at 14 and 28 DAF compared with the WT leaves (Figure 5A,B). A similar result was also observed with the MDA level in the flag leaves (Figure 5C). We also investigated ion leakage rates in the flag leaves. Consistently, SR displayed significantly lower ion leakage (Figure 5D), indicating that SR has less cell membrane damage during leaf senescence. Collectively, these data indicate that oxidative damage is reduced more in SR than in WT during senescence.

### 2.6. Elevated Activities of Ca^2+^-ATPase, Mg^2+^-ATPase, and Rubisco in Rice SR during Natural Senescence

As shown in Figure 6A,B, the activities of Ca^2+^-ATPase and Mg^2+^-ATPase in both SR and WT were decreased, but both activities were consistently higher in SR than in WT during natural senescence, with the maximum differences observed at 28 DAF, which suggested greater activity and stability of ATPases in SR compared with WT during natural senescence. Ribulose-1,5-bisphosphate carboxylase/oxygenase (Rubisco) is the predominant protein in photosynthesizing plant parts, which is degraded in leaves of intact plants during natural senescence [20]. During natural senescence, a severe reduction was detected in the activity of Rubisco in flag leaves detached from WT with time, whereas a minor reduction was measured in leaves of SR (Figure 6C). In addition, the Rubisco content in SR leaves was significantly higher than that in WT (Figure S2), which was consistent with Rubisco activity.

### 2.7. Enhanced Carbohydrate Assimilation in Rice SR

Previous TEM analysis revealed more and larger starch grains in MCs and BSCs and greater chloroplasts in BSCs of SR plants compared with WT (Figure 3G,H). To further assess the capacity of carbohydrate assimilation in SR, diurnal changes in starch and soluble sugar levels were measured in flag leaves at 7 DAF at 7:00, 12:00, and 17:00. As shown in Figure 7A, starch levels in flag leaves of SR were higher than those of WT throughout the day, with significant differences observed between 12:00 and 17:00. Furthermore, soluble sugar levels in SR were consistently higher than those in WT, with dramatic differences observed at all time points (Figure 7B). Overall, these results suggest that the capacity of carbohydrate assimilation is enhanced in SR.

RETRACTED

### 2.8. Large and Heavy Panicle in Rice SR

SR plants form larger panicles (Figure 8A). To quantify the grain yield of rice SR, a number of different measurements were made. The primary branches and secondary branches were 60.8% and 31.3% higher for SR panicles, respectively (Figure 8D,E). Furthermore, the grain number and weight per panicle of SR significantly increased by 61.2% and 56.0%, respectively (Figure 8B,E,F). However, the size of SR grains was reduced (Figure 8C), which was consistent with the decrease of 1000 grain weight (Figure 8G). This indicates that the introduction of exogenous sorghum DNA negatively regulates grain size and weight in rice. Unexpectedly, the seed yield per plant of SR plants was decreased by 16.6% compared with that of WT (Figure 8G), which was most directly related to the reduction of tiller number (Figure 2E). Although the introduction of exogenous sorghum DNA influences the balance between grain number and size in rice and results in a decrease in tillers, it has formed extralarge panicles and a significant increase in biomass.

## 3. Discussion

Engineering the C4 pathway into C3 crops is proposed to be an important way to improve radiation, nitrogen, water-use efficiencies, photosynthesis, and consequently crop yield [5,6]. However, the path to converting C3 plants into C4 is not yet fully elucidated after about nearly 30 years of efforts to install a C4 photosynthetic pathway into C3 plants. On the basis of the significant phenotypic changes in the transgenic rice SR (Figure 2), we hypothesized that the introduction of exogenous sorghum DNA could integrate some photosynthetic traits of sorghum into rice. In the present study, 174,529 high-quality reads were generated from the sorghum BTx623 genome by whole-genome resequencing of transgenic rice SR, and 71.21% reads were uniquely and confidently mapped to the sorghum genome, indicating that a few sorghum genes could be integrated into the rice genome by spike-stalk injection (Table S1, Figure 1). Previous studies experimentally confirmed that spike-stalk injection could integrate donor DNA fragments in the genomes of variants [19,20,21,22]. The spike-stalk injection method also caused extensive phenotypic and genotypic variations for rice by genomewide comparison [19]. In this study, four sorghum genes encoding C4 photosynthetic enzymes, including PEPC, PEPCK, PPDK, and NADP-ME, were selected for analysis. However, only the expression of *SbPEPCK* and *SbPPDK* was detected in SR (Figure 1B), suggesting that spike-stalk injection may not be able to integrate all C4 photosynthetic enzymes into rice. PPDK is the key enzyme for C4 photosynthesis in MCs. Conversely, in BCs, a high level of PEPCK is required for C4 acid [23]. PPDK acts in concert with PEPCK to catalyze the conversion of pyruvate to oxaloacetate, and that oxaloacetate can then be used to produce aspartate prior to the biosynthesis of transport amino acids [24].

RETRACTED

The current strategy for C4 rice is aimed at generating C4 photosynthesis with Kranz anatomy [25]. The critical initial step in all evolutionary trajectories from C3 to C4 was the transition from C3 to proto-Kranz [10,11,12]. Assessing the impact of exogenous sorghum DNA introduction on rice allowed for the investigation of the plasticity of rice leaves, specifically whether elements of Kranz anatomy can be introduced into them. In the present study, a comparative analysis of the leaf anatomy in both SR and its acceptor rice 9311 revealed that the introduction of exogenous sorghum DNA caused increases in leaf thickness (Figure 3F), bundle sheath (BS) number (Figure 3B−D) and size (Figure 3F), and size of chloroplasts in BSCs (Figure 3G), the key traits associated with proto-Kranz [5,26]. Increasing leaf thickness is an important approach to improve plant photosynthesis, for it leads to a greater number of mesophyll cells and higher carboxylation efficiency [27]. The increase in leaf thickness and BS size was likely to fulfil the requirements of C4 photosynthesis. Changes in leaf thickness will have consequences for the efficiency of light capture, which can also be affected by the different distributions of chloroplasts in MCs and BSCs [28]. Interestingly, the number of bundle sheaths was significantly increased, but the interbundle sheath distance was not decreased (Figure 3A−D). Collectively, these results demonstrate that the introduction of exogenous sorghum DNA to rice can induce the transition from C3 leaf anatomy to proto-Kranz.

Notably, the introduction of exogenous sorghum DNA into rice resulted in the improved photosynthesis and productivity of rice SR (Figure 2, Figure 4 and Figure 8). Enhanced photosynthetic efficiency together with delayed leaf senescence led to significantly increased accumulation of carbohydrates (both starch and sugars) and improved biomass and grain yields when SR was grown in the field. Additional lines of evidence indicated that these improvements were due to not only the photosynthetic CO_2_-concentrating effect but also an improvement in energy balance. (1) Compared with WT plants, SR plants displayed many additional phenotypes that are typical of CO_2_ enrichment, such as increases in the size of chloroplasts and starch grains, Chl contents, and carbohydrates (Figure 3, Figure 4 and Figure 7). (2) SR plants had growth advantages under higher light conditions, supported by the photosynthetic rate and light-response curves, and higher A_max_ and AQY observed for SR plants (Figure 4). (3) SR plants increased Rubisco content and activity, which enhanced carboxylation efficiency, CO_2_ fixation, and photosynthetic rate. A previous report indicated that the introduction of the small subunit (RbcS) of high catalytic turnover rate Rubisco from sorghum dramatically enhances the catalytic efficiency of Rubisco in transgenic rice [29]. However, Rubisco activation in transgenic lines was slightly decreased, and the capacity of electron transport was not sufficient to support the increased Rubisco capacity in transgenic rice, ultimately leading to no increase in photosynthetic rate [29]. Conversely, the present findings showed that the introduction of exogenous sorghum DNA into rice can not only increase the activity and content of Rubisco but also increase Ca^2+^ and Mg^2+^-ATPase activities for the demand of the capacity of higher RuBP carboxylation by Rubisco (Figure 6 and Figure S2). These results suggest that the exogenous sorghum DNA integration confers rice plant improved photosynthesis and productivity resulting from both photosynthetic CO_2_-concentrating effect and improved energy balance.

RETRACTED

We also observed that the introduction of exogenous sorghum DNA into rice resulted in delayed leaf senescence and was tightly linked to low accumulation of ROS and MDA, low electrolyte leakage, high Chl levels, and improved photosynthetic rate and biomass (Figure 2, Figure 3, Figure 4 and Figure 5). We speculate that higher photosynthesis and lower chloroplast degradation are the result of low ROS accumulation. The delayed leaf senescence can increase leaf longevity, which results in an increase in grain yield [30]. In previous reports, biomass and grain yields were not accounted for, although it was recently reported that a functional C4 metabolic pathway is achievable in rice [31]. Rice is the world’s most consumed crop, and increasing its grain yield is the ultimate objective. In the current study, increased photosynthesis and biomass yield could be stably detected for SR plants, but grain yield varied mainly depending on tiller numbers. A number of traits known to correlate with grain yield were markedly improved in SR plants, such as photosynthetic capability (Figure 4), aboveground biomass (Figure 2C−H), primary and secondary panicle branch numbers (Figure 8D,E), and grain number and weight per panicle (Figure 8F,G). However, the grain size and tiller numbers of SR were reduced (Figure 2E and Figure 8C), which directly led to a decrease in grain yield per plant. Therefore, one feasible approach to obtaining high yield is to increase the planting density of SR plants. Efforts are ongoing to reveal how exactly reduced tiller numbers occur in SR plants in order to overcome this flaw and maximize productivity.

In conclusion, our study presented one unique approach to engineering C4 rice that achieved the transition from C3 to proto-Kranz, and enhanced the productivity of transgenic rice resulting from both photosynthetic CO_2_-concentrating effect and improved energy balance. However, whether a functional C4 metabolic pathway is formed by spike-stalk injection in SR remains to be further studied.

## 4. Materials and Methods

### 4.1. Plant Materials and Growth Conditions

The transgenic plant sorghum–rice (SR) was generated via the spike-stalk injection method by inducing the total genome DNA of sorghum into a common *indica* rice cultivar 9311 (*Oryza sativa* L.) (wild type, WT) according to the protocol of Zhao et al. [18] and developed as a stable variant rice strain after six generations. All the experiments were conducted in two sets: one in the field and another in the pots. SR and the WT plants were grown in the field of Nanjing Normal University, China (32°10′ N, 118°91′ E), during the growing season from June to October. The seeds were germinated on filter paper moistened with water for 3 days at 30 °C after being sterilized with 30% H_2_O_2_ for 15 min. The germinated seeds were sown in a seedling nursery on May 1 and transplanted to pots filled with soil or field on 5 June. Pot planting was under natural conditions, and each pot contained three seedlings. Field planting was under natural conditions at a density of 20 × 30 cm per plant. The SR and WT plants were arranged in the field in a randomized block design with three replicates. Conventional agricultural management was carried out during the growing and developing of the seedlings.

### 4.2. DNA Extraction and Genome Resequencing

Genomic DNA was isolated from 20-day-old leaf tissue using a PureLink™ Genomic Plant DNA Purification Kit (Invitrogen, Carlsbad, CA, USA), according to the manufacturer’s specifications. The libraries were constructed with a TruSeq Nano DNA LT Sample Preparation Kit (Illumina, San Diego, CA, USA). Briefly, the genomic DNA was sheared into fragments with a length of ~350 bp using S220 Focused-ultrasonicators (Covaris, Woburn, MA, USA). Adapters were ligated onto the 3′ end of the sheared fragments. After PCR amplification and purification, the final libraries were sequenced on an Illumina sequencing platform HiSeq X Ten platform (Illumina, San Diego, CA, USA), and 150 bp paired-end reads were generated. The raw reads were subjected to a quality check and then filtered by fastp (version 0.19.5) [32]. Then, all clean reads were mapped with the genome sequences of *indica* rice R498 (http://mbkbase.org/R498, accessed on 3 January 2021) and sorghum BTx623 (https://phytozome.jgi.doe.gov, version 3.1.1, accessed on 3 January 2021) using a Burrows–Wheeler Aligner (BWA, version 0.7.12) [33]. After alignment, Picard (https://broadinstitute.github.io/picard, version 4.1.0.0, accessed on 8 January 2021) was employed to mark duplicate reads, and SAMtools (Version: 1.4) [34] was used to convert the alignment result format. The genome resequencing and analysis were conducted by OE Biotech Co., Ltd. (Shanghai, China). Raw sequence reads have been uploaded to the NCBI database (BioProject accession: PRJNA711573).

RETRACTED

### 4.3. RNA Extraction and Reverse Transcription Polymerase Chain Reaction (RT-PCR)

The total RNA from the seedling leaves of WT and SR was extracted with TRIzol (Invitrogen, Carlsbad, CA, USA). The quality and quantity of the purified RNA were assessed with a DS-11 spectrophotometer (DeNovix, Wilmington, DE, USA). A HiScript II RT Reagent Kit (Vazyme, Nanjing, China) was used to generate cDNA. RT-PCR was performed with a Veriti 96-Well Thermal Cycler (Applied Biosystems, Foster, CA, USA) according to the manufacturer’s instructions. The four sorghum genes encoding C4 photosynthetic enzymes, including phosphoenolpyruvate carboxylase (PEPC), phosphoenolpyruvate carboxykinase (PEPCK), pyruvate, orthophosphate dikinase (PPDK), and NADP-dependent malic enzyme (NADP-ME), were selected for analysis. The primers for RT-PCR were designed with the Primer Premier 5.0 software and are listed in Table S2.

### 4.4. Photosynthetic Measurements

Photosynthetic gas exchange measurements were carried out using a portable photosynthesis system (CIRAS-3, PP Systems, Amesbury, MA, USA). The fully expanded flag leaf on each plant from pot planting was used for the determination on sunny days. The net photosynthetic rates of SR and WT plants were generated under natural air and light conditions at 7 days after flowering (DAF), 14 DAF, and 28 DAF. For generation of the light-response curves, the conditions in the leaf chamber were set as follows: leaf temperature at 30 °C, CO_2_ concentration of 400 μmol mol^−1^, relative humidity at 70%, and gradually increasing PFD from 50 to 1800 μmol m^−2^ s^−1^ (controlled by a CIRAS-3 LED irradiation source). Light-response curves were fitted using the Farquhar–von Caemmerer–Berry model [35], and the light-saturated photosynthetic rate (A_max_) and apparent quantum yield (AQY) were calculated. The chlorophyll fluorescence was measured with a pocket chlorophyll fluorometer (Handy PEA, Hansatech, Kings Lynn, Norfolk, UK) between 9:30 and 10:30 on sunny days in uppermost, fully expanded flag leaves. The leaves were dark-adapted for at least 30 min before measurements. The professional PEA Plus and Biolyzer HP3 software were employed to calculate the maximal PSII quantum efficiency (F_v_/F_m_) and total performance index (PI_total_). Chlorophyll (Chl) was extracted from the fully expanded leaves with a mixed solution (45% acetone, 45% ethanol, and 10% distilled water), and the content was then determined by a spectrophotometer (GENESYS 10, Thermo Electron, Waltham, MA, USA) at 645 and 663 nm according to Lichtenthaler [36].

RETRACTED

### 4.5. Detection of Reactive Oxygen Species (ROS)

Leaf tissues of 0.5 g were homogenized in an ice bath in 5 mL of 65 mM phosphate buffer (pH 7.8) and centrifuged at 10,000 rpm for 15 min at 4 °C. The superoxide anion (O_2_^−^) was measured by monitoring nitrite formation from hydroxylamine following the method of Jiang et al. [37]. The mixture contained 200 μL supernatant, 750 μL phosphate buffer solution (65 mM, pH 7.8), 50 μL hydroxylamine hydrochloride (10 mM), 1 mL sulfanilamide (17 mM), and 1.0 mL α-naphthylamine (7 mM). The absorbance was measured at 530 nm, and a standard curve with NO_2_^−^ was used to estimate the production rate of O_2_^−^. Hydrogen peroxide (H_2_O_2_) was detected following the method of Jiang et al. [37]. The mixture contained 200 μL supernatant and 2 mL 20% H_2_SO_4_ (*v*/*v*) with 0.1% TiCl_4_ (*v*/*v*). The absorbance was measured at 410 nm, and the amount of H_2_O_2_ was extrapolated from the standard curve for H_2_O_2_.

### 4.6. Lipid Peroxidation and Electrolyte Leakage Determinations

Lipid peroxidation was estimated by determining the amount of malondialdehyde (MDA) produced by thiobarbituric acid (TBA) reaction according to the method of Draper and Hadley [38]. For this, leaf samples (0.5 g) were homogenized in 5 mL of 0.1% trichloroacetic acid (TCA) and centrifuged at 10,000 rpm for 10 min at 4 °C. The supernatant was used to assay for MDA concentration. The electrolyte leakage percentage (%) was measured as described previously [39] with minor modifications. Briefly, the fresh leaves were cut into 1 cm slices and washed twice with distilled water, and then transferred into a glass test tube with 20 mL distilled water for 2 h at 28 °C. At this time, the conductivity of the solution was measured as the initial electrical conductance (EC1). EC2 was measured after boiling samples for 30 min. Electrolyte leakage was quantified using the following equation: electrolyte leakage (%) = (EC1/EC2) × 100.

RETRACTED

### 4.7. Starch and Soluble Sugar Content Measurements

Starch and soluble sugar were extracted from rice leaves and measured by the anthrone reaction as described previously [40] with slight modifications. Briefly, the leaves were dried at 75 °C until the mass maintained stability. The dried samples were ground to powder, and then soluble sugar was extracted twice with 5 mL of 80% ethanol at room temperature. The remaining samples were further washed three times with 5 mL of 80% ethanol and twice with 5 mL of distilled H_2_O_2_. Starch was then extracted with HClO_4_ (29% *v*/*v*) at 4 °C. The soluble sugar content of the samples was measured at 630 nm after the reaction with anthrone–sulfuric acid reagent (100 °C, 10 min) using glucose as a standard. Soluble sugar content was expressed as glucose equivalents, and starch content was calculated by multiplying the equivalents by 0.90.

### 4.8. Ca^2+^-ATPase, Mg^2+^-ATPase, and Rubisco Activity Determinations

Chloroplasts were isolated from leaves following the procedure of Kügler et al. [41]. Briefly, the leaves (2 g) were homogenized in 20 mL ice-cold isolation buffer containing 30 mM HEPES (pH 7.8), 2 mM EDTA, 0.1% BSA (*w*/*v*), 330 mM mannitol, and 3 mM MgCl_2_. All subsequent steps were carried out at 4 °C. The homogenate was filtered through four layers of muslin and centrifuged at 2000× *g* at 4 °C for 5 min. The chloroplasts were further purified by gradient centrifugation in 10 mL extraction buffer containing 40% Percoll at 30,000× *g* for 30 min. Ca^2+^-ATPase and Mg^2+^-ATPase activities were assayed according to the method of Wang et al. [42]. For the measurement of Ca^2+^-ATPase activity, the chloroplast suspension (1 mL) was added to 1 mL reaction solution containing 250 mM tricine (pH 8.0), 10 mM ATP, 20 mM EDTA, and 0.2% trypsin (*w*/*v*), and incubated at 20 °C for 10 min. Then, 0.1 mL 1% BSA was added to the mixture to terminate the reaction. An amount of 0.5 mL of the incubated chloroplast suspension was added to 0.5 mL of the reaction mixture containing 0.5 M tricine (pH 8.0), 50 mM CaCl_2_, and 10 mM ATP. The mixture was incubated at 37 °C for 10 min and centrifuged at 3000× *g* for 1 min, and the supernatant was used to determine the content of inorganic phosphorus. For the measurement of Mg^2+^-ATPase activity, the chloroplast suspension (1 mL) was added to 1 mL reaction solution containing 250 mM tricine (pH 7.0), 0.5 M NaCl, 50 mM DTT, and 50 mM MgCl_2_, and incubated in high irradiance at 25 °C for 5 min. Then, 0.1 mL 1% BSA was added to the mixture to terminate the reaction. An amount of 0.5 mL of the incubated chloroplast suspension was added to 0.5 mL of the reaction mixture containing 0.5 M tricine (pH 8.0), 50 mM CaCl_2_, and 50 mM ATP. The mixture was incubated at 37 °C for 10 min and centrifuged at 3000× *g* for 1 min, and the supernatant was used to determine the content of inorganic phosphorus. Rubisco activity was determined according to Bota et al. [43]. The leaves were homogenized in 1 mL of an ice-cold extraction medium containing 0.1 m bicine (pH 8.0), 2 mM benzamidine, 50 mM β-mercaptoethanol, 6% PEG 4000, 20 mM MgCl_2_, 11 mM Na-diethyl-dithio-carbamate, 2 mM ε-amino-n-caproic acid, 2 mM phenylmethylsulfonyl fluoride, 1% (*v*/*v*) protease inhibitor cocktail, and 2.5% Tween 20. Extracts were centrifuged at 12,000 rpm for 2 min at 4 °C, and the resulting supernatant immediately assayed at 25 °C for Rubisco activity. The initial and total activities were determined according to Parry et al. [44].

RETRACTED

### 4.9. Immunoblot Analysis

SDS-PAGE and immunoblot analysis of the Rubisco protein were performed as described in Balasaheb et al. [45]. Briefly, leaf tissues were ground in liquid nitrogen and then homogenized with sample buffer (50 mM tris, pH 6.8; 10% glycerol; 2% SDS; 2 mM EDTA; and 6% 2-mercaptoethanol). Homogenates were centrifuged at 12,000 rpm for 3 min, and supernatants were denatured at 90 °C for 5 min. Aliquots of the leaf protein extracts were subjected to 12% (*w*/*v*) SDS-PAGE, and resolved proteins were transferred onto a polyvinylidene difluoride (PVDF) membrane (Bio-Rad, Bedford, MA, USA). Antibody against Rubisco large chain (RbcL, Agrisera, Vännäs, Sweden) was used for immunoblot analysis. The protein levels were detected using an enhanced chemiluminescence detection reagent (High-sig ECL, Tanon, Shanghai, China) according to the manufacturer’s instructions.

### 4.10. Transmission Electron Microscopy (TEM)

Fresh leaf tissue for the TEM analysis was harvested from the plants in the paddy fields at 7 DAF. The detached leaves were soaked in a fixation buffer (2% glutaraldehyde in 0.1 M phosphate buffer, pH 7.2) under vacuum and postfixed for 4 h in phosphate-buffered saline containing 2% OsO_4_ (pH 7.2), transferred back into phosphate buffer, and washed several times. After dehydration through an acetone series, samples were embedded in LR white resin (London Resin, Berkshire). Ultrathin sections were cut using a diamond knife on a Leica EMUC6 microtome, then double-stained with 2% (*w*/*v*) uranyl acetate and 2.5% (*w*/*v*) lead citrate aqueous solution. The prepared samples were observed under a Hitachi 600A-2 (Japan) TEM.

RETRACTED

### 4.11. Statistical Analysis

All experiments were repeated independently for at least three replicates, and data were subjected to statistical analysis using Student’s *t*-test with a *p*-value less than 0.05 considered significant.

## Figures and Tables

**Figure 1:** Genomewide distribution (**A**). The *x*-axis represents the chromosome position. The *y*-axis indicates the average coverage reads. (**B**) Total RNA extracted from leaves of WT and SR was used for RT-PCR analysis with gene-specific primers as listed in Table S2.

**Figure 2:** Characteristics of wild type (WT) and transgenic plant sorghum–rice (SR). (**A**) Phenotypes of WT (left) and SR (right) at 21 days after flowering (DAF). Bars, 20 cm. (**B**) Magnified views of a flag leaf taken 7 DAF from WT (left) and SR (right). Bar, 5 cm. (**C**–**H**) Increased vegetative biomass in SR. Plant height (**C**), total dry weight per plant (**D**), tiller number (**E**), flag leaf length (**F**), flag leaf width (**G**), and flag leaf area (**H**) of WT and SR. Values (**C**–**H**) are given as means ± SD (*n* ≥ 15). Asterisks indicate significant differences between WT and SR. ** *p* < 0.01 compared with WT by Student’s *t*-test.

**Figure 3:** Comparing wild-type (WT) and transgenic plant sorghum-rice (SR) flag leaf phenotypes at 7 days after flowering (DAF). (**A**) Segregant leaf surface of WT (top) and SR (bottom). Bar, 5 mm. (**B**) Large bundle sheath number of WT and SR. (**C**) Small bundle sheath number of WT and SR. (**D**) Total bundle sheath number of WT and SR. (**E**) Interbundle sheath distance of WT and SR. (**F**) Flag leaf cross sections of WT (left) and SR (right) plants at 28 DAF. LBS, large bundle sheath; SBS, small bundle sheath; BSC, bundle sheath cell; MC, mesophyll cell. Bar, 100 μm. (**G**,**H**) Transmission electron micrographs of leaf sections showing bundle sheath cells and mesophyll cells from WT (top) and SR (bottom) at 14 DAF. Ch, chloroplast; ST, stromal thylakoid; GT, grana thylakoid; SG, starch grain; P, plastoglobule. Bars, 1 μm. Values (**B**–**E**) are given as means ± SD (*n* = 10). Asterisks indicate significant differences between WT and SR. ** *p* < 0.01 compared with WT by Student’s *t*-test.

**Figure 4:** SR exhibits a higher rate of photosynthesis than WT. (**A**) Light-response curves of flag leaves in WT and SR were generated at 7 DAF at a temperature of 30 °C under normal air conditions. (**B**,**C**) A_max_ (light-saturated photosynthetic rate) and AQY (apparent quantum yield) of flag leaves in WT and SR were calculated from the light-response curves. (**D**) Total Chl level of flag leaves in WT and SR. FW, fresh weight. (**E**) Photosynthetic rates of WT and SR. Flag leaves were consistently measured under normal air conditions. (**F**,**G**) F_v_/F_m_ (maximal PSII quantum efficiency) and PI_total_ (total performance index) of flag leaves in WT and SR. Values (**B**,**C**) are given as means ± SD (*n* = 3). Value (**D**) is given as mean ± SD (*n* ≥ 6). Values (**E**–**G**) are given as means ± SD (*n* ≥ 6). Asterisks indicate significant differences between WT and SR. * *p* < 0.05; ** *p* < 0.01 compared with WT by Student’s *t*-test.

RETRACTED

**Figure 5:** SR exhibits reduced ROS accumulation and oxidative damage in leaves during senescence. (**A**) O_2_^–^ content of flag leaves in WT and SR. (**B**) H_2_O_2_ content of flag leaves in WT and SR. (**C**) MDA content of flag leaves in WT and SR. (**D**) Electrolyte leakage of flag leaves in WT and SR. Values (**A**–**D**) are given as means ± SD (*n* = 3). Asterisks indicate significant differences between WT and SR. * *p* < 0.05; ** *p* < 0.01 compared with WT by Student’s *t*-test.

**Figure 6:** Higher activities of Ca^2+^-ATPase, Mg^2+^-ATPase, and Rubisco and content of Rubisco in SR during senescence. (**A**–**C**) Ca^2+^-ATPase (**A**), Mg^2+^-ATPase (**B**), and Rubisco (**C**) activities of WT and SR. Values (**A**–**C**) are given as means ± SD (*n* = 3). Asterisks indicate significant differences between WT and SR. * *p* < 0.05; ** *p* < 0.01 compared with WT by Student’s *t*-test.

**Figure 7:** Leaves of SR accumulate significantly higher levels of starch and soluble sugar than WT. (**A**,**B**) Starch (**A**) and soluble sugar (**B**) levels measured in flag leaves at 7 DAF at 7:00, 12:00, and 17:00. Values (**A**,**B**) are given as means ± SD (*n* = 6). Asterisks indicate significant differences between WT and SR. * *p* < 0.05; ** *p* < 0.01 compared with WT by Student’s *t*-test.

**Figure 8:** SR forms large and heavy panicle. (**A**) Representative photograph of panicle morphology of SR plant. Bar, 5 cm. (**B**) Seed yield per panicle of WT and SR. Bars, 2 cm. (**C**) Mature paddy (top) and brown (bottom) rice grains of WT and SR. Bars, 1 cm. (**D**) Number of WT and SR primary panicle branches. (**E**) Number of WT and SR secondary panicle branches. (**F**) Grain number per panicle of WT and SR. (**G**) Grain weight per panicle of WT and SR. (**H**) 1000 grain weight of WT and SR. (**I**) Seed yield per plant of WT and SR. Values (**D**–**I**) are given as means ± SD (*n* ≥ 15). ** *p* < 0.01 compared with the WT by Student’s *t*-test.

RETRACTED

## Data Availability

The original contributions presented in the study are publicly available. These data can be found here: https://www.ncbi.nlm.nih.gov/bioproject/PRJNA711573 (accessed on 10 March 2021).

## Supplementary Materials

The following are available online at https://www.mdpi.com/article/10.3390/ijms22094305/s1.
